# Automated Screening of COVID-19-Based Tongue Image on Chinese Medicine

**DOI:** 10.1155/2022/6825576

**Published:** 2022-06-23

**Authors:** Guang Zhang, Xueying He, Delin Li, Cuihuan Tian, Benzheng Wei

**Affiliations:** ^1^School of Software, Shandong University, Jinan 250101, China; ^2^Health Management, The First Affiliated Hospital of Shangdong First Medical University & Shandong Provincial Qianfoshan Hospital, Jinan 250014, China; ^3^College of Intelligence and Information Engineering, Shandong University of Traditional Chinese Medicine, Jinan 250355, China; ^4^School of Medicine, Shandong University, Jinan 250012, China; ^5^Health Management Center, Qilu Hospital of Shandong University, Jinan 250012, China; ^6^Center for Medical Artificial Intelligence, Shandong University of Traditional Chinese Medicine, Qingdao 266112, China

## Abstract

**Objective:**

Artificial intelligence-powered screening systems of coronavirus disease 2019 (COVID-19) are urgently demanding since the ongoing outbreak of SARS-CoV-2 worldwide. Chest CT or X-ray is not sufficient to support the large-scale screening of COVID-19 because mildly-infected patients do not have imaging features on these images. Therefore, it is imperative to exploit supplementary medical imaging strategies. Traditional Chinese medicine has played an essential role in the fight against COVID-19.

**Methods:**

In this paper, we conduct two kinds of verification experiments based on a newly-collected multi-modality dataset, which consists of three types of modalities: tongue images, chest CT scans, and X-ray images. First, we study a binary classification experiment on tongue images to verify the discriminative ability between COVID-19 and non-COVID-19. Second, we design extensive multimodality experiments to validate whether introducing tongue image can improve the screening accuracy of COVID-19 based on chest CT or X-ray images.

**Results:**

Tongue image screening of COVID-19 showed that the accuracy (ACC), sensitivity (SEN), specificity (SPEC), and Matthew correlation coefficient (MCC) of the improved AlexNet and Googlenet both reached 98.39%, 98.97%, 96.67%, and 99.11%. The fusion of chest CT and tongue images used a tandem multimodal classifier fusion strategy to achieve optimal classification, and the results and screening accuracy of COVID-19 reached 98.98%, resulting in a significant improvement of 4.75% the highest accuracy in 375 years compared with the single-modality model. The fusion of chest x-rays and tongue images also had good classification accuracy.

**Conclusions:**

Both experimental results demonstrate that tongue image not only has an excellent discriminative ability for screening COVID-19 but also can improve the screening accuracy based on chest CT or X-rays. To the best of our knowledge, it is the first work that verifies the effectiveness of tongue image on screening COVID-19. This paper provides a new perspective and a novel solution that contributes to large-scale screening toward fast stopping the pandemic of COVID-19.

## 1. Introduction

With the pandemic of coronavirus disease 2019 (COVID-19) worldwide, the automated system is significantly urgent and necessary to realize large-scale screening. COVID-19 is a respiratory infectious disease caused by the novel virus named severe acute respiratory syndrome coronavirus 2 (SARS-CoV-2). SARS-CoV-2 has so high human-to-human transmission ability that it seriously threatens the health of people around the world. According to the World Health Organization (WHO), until April 29, 2022, more than 511,234,994 people have suffered from COVID-19 worldwide to date. Among them, more than 6,255,880 people have died. With the rapid increase of COVID-19 cases every day, fast and large-scale screenings are imperative to cut off the source of infection. Although nucleic acid detection is the gold standard in clinical, the availability, stability, and reproducibility of nucleic acid detection kits are problematic [1, 2]. Nowadays, medical imaging examinations, such as chest computed tomography (CT) and X-ray, play an essential role in the screening process of COVID-19. However, medical imaging-based screening of COVID-19 is under problem with enormous pressure in clinical, i.e., the rapidly growing amount of COVID-19 cases makes global medical resources unbearable [3, 4]. Automated screening systems of COVID-19 can correspondingly assist the clinical practice in accelerating the large-scale screening and alleviating the global shortage of medical supplies. Therefore, it is significantly urgent and necessary to study on automated screening systems.

In practice, a new supplementary examination approach is demanding to improve the screening accuracy and reduce the radiation dose. While a few recent studies on automated COVID-19 screening have made great progress, they only focus on designing either chest CT-based approaches or X-ray-based techniques [1, 2, 4–21]. Both chest CT and X-ray are common medical imaging methods in clinical but have three-fold limitations in the task of automated screening of COVID-19. First, they cannot present imaging features for mild infected cases, such that it is impossible to screen mild COVID-19 patient [22, 23]. Second, existing studies have indicated that the accuracy rates of existing methods are not too satisfied, and the single-modality data alone is not sufficient to support real-world clinical applications [3]. Finally, the CT and X-ray examinations are not easily accessible, and their radiation doses are very high.

In the global fight against COVID-19, tongue image analysis contributes to the diagnosis and treatment in clinical. Tongue image plays a vital role because it has many advantages, such as light, quick, and availability. Analyzing tongue images is an efficient strategy and the foundation of traditional Chinese medicine (TCM) in the COVID-19 diagnosis clinically. Tongue images carry special features of COVID-19 and thus can provide relevant references for TCM, which has successfully accelerated the recovery of COVID-19 patients and reduced the use of antibiotics in China [24, 25]. According to the clinical analysis of TCM, the main manifested characteristics of COVID-19 in tongue images are the tongue color, the thickness of tongue coating, the degree of greasy coating, and the cracks of the tongue body. Interestingly, the tongue color changes of mild COVID-19 patients are noticeable, making up the lack of CT and X-ray. Thus, tongue images provide another diagnostic approach for people who do not have visible radiographic features with mild or asymptomatic infection. On the other hand, the imaging devices of tongue images are easily accessible, light, and quick. In case of emergency, COVID-19 patients can use the mobile phone or digital camera to take the tongue image and send it to remote doctors without touch, preventing the spread of the virus.

In this paper, we investigate to answer a widely concerning question: can tongue image assist the automated screening of COVID-19? To examine the role of tongue image, we collected a real-world multimodality dataset from clinical. This dataset consists of three types of modalities: tongue images, chest CT scans, and X-ray images. Based on this dataset, we conduct extensive verification experiments in terms of two aspects. First, we design a binary classification experiment on tongue images to verify whether tongue images can discriminate COVID-19 and non-COVID-19. Second, we develop comprehensive multimodality analyses to validate whether combining tongue images with chest CT or X-rays can improve the screening accuracy of COVID-19. Theoretically, introducing the information of tongue images will be more helpful in identifying COVID-19. Therefore, we adopt dual-stream feature fusion networks to verify further whether adding tongue image features can help improve the screening accuracy of COVID-19. Both the two aspects' experimental results demonstrate that tongue image not only has an excellent discriminative ability for screening COVID-19 but also enhances the screening accuracy. To the best of our knowledge, it is the first work that verifies the effectiveness of tongue image on screening COVID-19. This paper provides a new perspective and a novel solution toward fast stopping the widespread of COVID-19. From another point of view, this paper demonstrates the importance of integrating Chinese and western medicine to diagnose COVID-19 in clinical.

The significant contributions of this paper include as follows:

- In this study, we verify the role of tongue image in the emerging task of COVID-19 screening. Our results have demonstrated the discriminative ability of tongue image
- In this study, we achieve multimodality image-based screening of COVID-19, which paves a reliable way for future studies in the medical image analysis community
- In this study, we demonstrate the feasibility and effectiveness of information fusion between tongue image and other medical images and provide a novel screening solution for the COVID-19 in clinical

## 2. Related Work

This section presents related works in terms of automated screening of COVID-19, multimodality methods, and tongue image-based methods in the medical image analysis community.

### 2.1. Automated Screening of COVID-19

To join in the global fight against COVID-19, lots of emerging works devoted to designing automated technologies for improving the clinical diagnostic efficiency, including automated screening [1, 2, 5–11], patient severity assessment [26], infection quantification [27], and infection area segmentation [8, 28]. While existing screening works of COVID-19 have achieved promising performance, to the best of our knowledge, no work has achieved automated analysis of COVID-19 based on tongue images. Among them, automated screening of COVID-19 received the most attention, involving chest CT- or X-ray-based works.

#### 2.1.1. CT-Based Screening of COVID-19

Since chest CT is the most-widely used imaging examination in clinical, a large part of studies focus on CT-based screening of COVID-19, including lesion patch-based methods [1, 2, 5, 6], 2D slice-based methods [7–10], and 3D scan-based methods [3, 11]. First, lesion patch-based approaches either need lesion annotations or are prone to errors from intermediate steps. For example, Wang et al. [1] firstly used a threshold approach to extract ROI (region of interest) patches and then trained a modified inception network to screen COVID-19 from typical 105 viral pneumonia. They collected chest CT scans from 79 cases of COVID-19 and 180 cases of typical viral pneumonia with 79.3% accuracy. Based on a large-scale dataset, Shi et al. [5] firstly trained a VB-Net to segment ROIs and then extracted manually-designed features to fit a random forest on classifying COVID-19 and common pneumonia. Second, the slice-based methods need the manual selection of slices to train the classifier, and they neglect the spatial correlation in CT scans, which is the key for the screening of COVID-19. For instance, Gozes et al. [8] used a 2D CNN to perform slice-level classification on 270 slices comprised of 120 COVID-19 and 150 normal slices. Finally, 3D scan-based methods can achieve optimal minima by leveraging end-to-end optimization, which often obtains better performance than multistage methods. For instance, Zhongyi et al. [3] formulated the 3D CT screening task as the problem of multiple instance learning and proposed a novel approach of attention-based deep 3D multiple instance learning, which achieves accurate and interpretable screening of COVID-19.

#### 2.1.2. X-Ray-Based Screening of COVID-19

Since regular X-ray machines are easily accessed in most primary hospitals where CT scanners are insufficient, X-ray based method is urgently needed. Based on public chest X-ray data, Li et al. [4] proposed a discriminative cost-sensitive learning approach to address the new problem of automated screening of COVID-19. Hassanien et al. [29] used a multilevel threshold segmentation algorithm to crop lung areas and adopted SVM to classify COVID-19 and normal cases based on 40 chest X-rays. Ozturk et al. [30] ensembled several feature extraction algorithms and used a stacked autoencoder with principal component analysis to make decisions. They showed that handcrafted feature-based classifiers perform better than deep models on small data. Several studies applied popular deep learning techniques for the screening of COVID-19. Hemdan et al. [31] validated the effectiveness of multiple popular deep models based on X-ray datasets.

### 2.2. Multimodality Fusion

Multimodality data can introduce comprehensive useful information and provide more distinct views. Generalized multimodality learning methods always extract and fuse information from multiple heterogeneous sources simultaneously. Prominent theoretical advance and effective algorithm have been achieved in the medical image analysis community. To achieve the accurate classification of chest diseases, Wang et al. [32] proposed the Text-Image Embedding Network that conducts the fusion of two heterogeneous sources comprised of medical records and medical images. This method gains a significant improvement compared to single-modality data. Zhou et al. [33] and Zhou et al. [34] made maximum use of four types of heterogeneous data (image, gene, etc.) to diagnose Alzheimer's disease (AD). Their experimental results show that AD diagnosis's accuracy can be significantly improved when using these multimodality data simultaneously.

On the other hand, narrow multimodality data is always one type of specific medical image generated by different imaging principles. The narrow multimodality data can present the same anatomical structure from different views. For example, Liu et al. [35] proposed a fusion network to combine magnetic resonance imaging (MRI) images and positron emission tomography (PET) images. This work achieved satisfactory classification performance in the task of AD analysis. Li et al. [36] proposed the HyperDenseNet that combines CT and MRI images to perform the segmentation of lung tumors. The comparison between related works of AI-based COVID-19 analysis is shown in Table 1. This work also made a significant improvement. In this paper, our objective is to fuse tongue images and radiology images to validate the role of tongue images for finding a new solution and realize the accurate screening of COVID-19.

### 2.3. Tongue Image Analysis

Tongue diagnosis is an important and dominant part of TCM computer-aided diagnosis and treatment [37]. With the advancement of the tongue meter, the tongue image can be a high-quality record of tongue color, water, grease, depressions, fissures, and much other valuable information of concern to Chinese medicine [38]. Accurate segmentation and appropriate feature extraction are the heart of automated tongue diagnosis. Zhou et al. [39] proposed a TongueNet for the tongue image segmentation. TongueNet derives from U-Net and adds a morphological layer at the top of the network structure, which achieved the highest segmentation result with a pixel-level accuracy of 98.45%. Zeng et al. [40] proposed the Boundary Guidance Hierarchical Network (BGHNet) and achieved an end-to-end optimization for mixed losses. Srividhya and Muthukumaravel [41] combined the extracted features and texture analysis results to train support vector machines (SVM) for the classification of tongue images. Yousif and Saud [42] used Gabor filters to extract representative features and obtained promising results on tongue image analysis.

The most representative work is achieved by Wu et al. [43], who presented a conformal mapping method for tongue image alignment. This method has a strong ability to resist tongue deformation. At the same time, this work realized automated analyses of 10 types of diseases, including but not limited to diabetes, fatty liver, lung cancer, and breast cancer. While prominent works have achieved promising progress, no work has achieved the automated analysis of COVID-19 based on tongue images. In this paper, we validate the effectiveness of tongue images on the screening task of COVID-19.

## 3. Materials and Methods

In this section, we introduce the newly-collected multimodality dataset comprised of tongue images, chest CT, and X-rays. Then, we describe how the collected dataset is processed in the experiments. Finally, we give the full details of the methodology employed in this study, including a single-modality model and a multimodality information fusion model.

### 3.1. Dataset

In this study, we collected a multimodality dataset from COVID-19 designated treatment hospitals in Shandong Province. This dataset consists of three types of modalities, and the randomly-selected samples are illustrated in Figure 1. This dataset includes 488 patients comprised of 188 COVID-19 patients and 300 non-COVID-19 patients. This study and all research were approved and conducted following relevant guidelines/regulations. Moreover, the degree of severity is divided into mild, ordinary, severe, and critical according to clinical standard. Without loss of generality, the non-COVID-19 patients are healthy or have other diseases, such as common viral pneumonia and bacterial pneumonia. Every COVID-19 patient was confirmed with nucleic acid detection kits of reverse transcription-polymerase chain reaction (RT-PCR).

Since each patient has been tested several times, the data from the same patient have at least two days gap to ensure diversity. The splitting of the data is according to the patient level, i.e., no data from the same patient exists in training and testing sets, simultaneously. Figures 2 and 3 present the patient number and image number of the training set, validation set, and test set among the three modalities, respectively. In the test set, the severity degrees of COVID-19 patients are shown in Figure 4. We can see that the ordinary degree among the 17 COVID-19 patients accounts for the majority. Note the time interval between the acquisition of the X-rays/CT image and the tongue image not exceeding 24 hours.

When training, data augmentation strategies include radiation transformation and color dithering. Specifically, the radiation transformation includes random rotation (0 ± 30) and horizontal flips. The color dithering includes accidental adjustment of brightness (0% ± 50%) and contrast (0% ± 30%). Besides, we normalized all images to reduce the impact of different imaging devices on the data distribution.

### 3.2. Single-Modality Model

We use the common AlexNet as the backbone for the screening of COVID-19 based on single-modality data. The original AlexNet has eight layers, which include five convolutional layers and three pooling layers. The convolutional layers used a 11 × 11 filter, a 5 × 5 filter, and three 3 × 3 filters. Three max-pooling layers with 2 × 2 kernel are deployed after the first, second, and fifth convolutional layers. We set the output shape of the last convolutional layer's features to be 6 × 6 × 512 and flatten them. The original fully connected layers of AlexNet are removed and replaced by two trainable fully-connected layers. The channel numbers of the two fully-connected layers are 64 and 2, respectively. The network structure of the modified AlexNet is shown in Table 2. Since the collected dataset is too small to obtain promising results through training the AlexNet from scratch, we use a transfer learning strategy. The parameters of the convolutional layers are initialized from the pretrained model based on ImageNet.

### 3.3. Multimodality Feature Fusion Model

The single modality of chest CT or X-ray is not sufficient to support the large-scale screening of COVID-19. The reason is that the patients with mild type do not have imaging features on chest CT or X-ray, resulting in a high misdiagnosis rate. To combine the imaging features from tongue images, we design a multimodality feature fusion model for extracting and fusing the semantic elements from different modalities.

As shown in Figure 5, the multimodality feature fusion model has three subtle modules. First, a feature extraction module is designed to generate deep heterogeneous features. This module has dual paths that extract features from two different modalities. Among them, each path has the same structure as the single-modality model. Each path will generate a 64-D feature vector. During the training phase, the two paths will be jointly optimized. Second, a fusion layer is proposed for integrating the deep heterogeneous features. Finally, a classifier module is deployed on the fused features for performing the final prediction. The classifier module is comprised of two fully connected layers. In the following content, we introduce the fusion layer comprehensively.

The fusion layer is the essence of the multimodality feature fusion model. To better check the feasibility of tongue images, we design three types of fusion strategies. The first fusion strategy is concatenation, which connects two feature vectors [44]. Assume the dimensions of two feature vectors are *P* and *Q*, respectively. The size of the fused feature vector is *P* + *Q*. The concatenation fusion strategy can keep the raw representative information of specific modality data, which could efficiently test the semantic ability of the extracted feature from tongue images. The second fusion strategy is the addition operation, which adds two feature vectors point-to-point. The addition fusion strategy requires that the input feature vectors have the same dimension [45]. Assume the dimensions of two feature vectors are *P* and *Q*, where *P* = *Q*. The dimension of the fused feature is *P*. The advantage of the addition fusion strategy is that the different features can be thoroughly fused to eliminate unilateral effects.

The final fusion strategy is the attention gate (AG) module proposed by Schlemper et al. [46]. The schematic of the AG module is shown in Figure 6. After adding the feature vectors generated by the two backbone networks, a 1 × 1 convolution layer with Softmax function is adopted. Then, the spatial region is selected by analyzing the activated context information. The trilinear interpolation method is adopted to resample the attention coefficient. The resampled coefficients are multiplied on the raw feature vector. Finally, we flatten the multiplied feature vector to obtain the fused feature vector. The AG module can generate a semantic and useful representation for multimodality data and usually achieve better performance. These three information fusion strategies can analyze the impact of the introduction of tongue images from different perspectives. The feasibility of tongue images can be fully demonstrated.

## 4. Results and Discussion

We verify tongue images on the newly-collected multimodality dataset using state-of-the-art algorithms. The code and dataset will be publicly available. In this section, we introduce the set-up of experiments, then present the binary classification results of the tongue images and the multimodality classification results of COVID-19 to demonstrate the feasibility of tongue images on the screening task of COVID-19. We finally give in-depth analyses in terms of noisy robustness and *t*-test.

### 4.1. Set-Up

#### 4.1.1. Tasks

We conduct two screening tasks for better verifying the tongue images in the problem of COVID-19 screening. The first task is the screening of COVID-19 based on tongue images. The positive class is COVID-19, and the negative class is non-COVID-19. From the practical point of view, the non-COVID-19 CT scans involve both common pneumonia and no pneumonia. The second task is the screening of COVID-19 based on three types of modalities data: tongue images, chest X-rays, and chest CT. Among the second task, we first combine tongue images and chest X-rays to screen COVID-19 for verifying whether or not using tongue images can improve the screening accuracy based on chest X-rays alone. We then combine tongue images, and chest CT for ascertaining whether or not using tongue images can enhance the screening accuracy based on chest CT alone. The split of data is according to the patient level.

#### 4.1.2. Configurations

In order to verify the effectiveness of tongue images, we compare various state-of-the-art methods: VGG19 [47], GoogLeNet [48], ResNet18 [49], ResNet50 [50], DenseNet [51], and the modified AlexNet for the first task. We compare three types of feature fusion approaches: concatenate, add, and attention gate for the second task. We also report the screening results of COVID-19 based on chest CT or X-rays, respectively. We implement our algorithm in Pytorch. Adam optimizer is used with an initial learning rate of 1*e* − 4 and other default parameters, following a training strategy that reduces the learning rate by 0.1 times every ten epochs. The input shape is 256 × 256. We set the training epoch *T* to 40 and the batch size to 32. All classifiers are deployed in the large server that includes an Nvidia GPU Tesla V100 GPU with cuDNN v9.0 and an Intel CPU Xeon(R) Gold 6246@3.30 GHz. All the compared models are implemented according to their open-source codes.

#### 4.1.3. Evaluation Metrics

The evaluation metrics include accuracy (ACC.), sensitivity (SEN.), specificity (SPEC.), Matthew correlation coefficient (MCC), the area under curves (AUC), and confusion matrix. Sensitivity measures the proportion of correctly identified positive data (i.e., COVID-19), and specificity measures the percentage of correctly identified negative data. The AUC value is an index that measures the entire two-dimensional area underneath the entire receiver operating characteristic (ROC) curve. The confusion matrix is a table with two rows and two columns that reports the number of false positives, false negatives, true positives, and true negatives. We also report the ROC curves for better analyzing the screening performance of tongue images.

### 4.2. Screening Result of COVID-19 Based on Tongue Images

To verify the ability of tongue image in the automated screening of COVID-19, we carried out a large number of experiments based on tongue images using three types of deep learning classification models.  Table 3 reports the results on the screening of COVID-19 based on tongue images. All the implemented algorithms are achieving promising performance. For example, both the modified AlexNet and GoogLeNet obtain the same state-of-the-art performance with a classification accuracy of 98.39%, a sensitivity of 98.97%, a specificity of 96.67%, and Matthew correlation coefficient of 99.11%. Saygl proposed a method based on image processing and machine learning to automatically detect viruses through segmented CT images with optimal accuracy values of 98.5% in dataset 1, 86.3% in dataset 2, and 94.5% in mixed dataset [18]. The screening results of other algorithms also remarkably outperform 90% on all the metrics. These rigorous results demonstrate that tongue images have the discriminative ability to screen COVID-19, which positively answers the question that tongue image can assist in the automated screening of COVID-19. Note that the modified AlexNet has fewer parameters and faster convergence. Therefore, the modified AlexNet is capable of the basic model of the multimodality networks. As shown in Figure 1, even the features of mild COVID-19 patients are unobvious, and the indiscernible infection areas lead to unusual difficulties; using tongue images still obtains accurate performance, which demonstrates the generalization and robustness under challenging environments.

Figure 7 shows the confusion matrix of the COVID-19 screening based on tongue images using the modified AlexNet. Our algorithm obtains a balance performance. From another view, these results demonstrate that the characteristic features of COVID-19 on tongue images are different from non-COVID-19. Therefore, they are easy to be distinguished by deep models. After revisiting the bad cases, we found that the misclassified images are belonging to ordinary COVID-19 patients. The reason is that the misclassified tongue images are ruddy, white, and unobvious greasy due to the light. This analysis indicates that although the collection of tongue images is convenient, the imaging conditions are strict, and the development of collection standards is urgently required.

### 4.3. Screening Result of COVID-19 Based on Multimodality Data

This section aims to verify whether or not introducing tongues images can improve the screening accuracy of COVID-19. As a baseline, we first implemented a single-modality model for the screening of COVID-19 based on single-modality data: chest CT or X-rays. We then use the newly-designed dual-stream neural networks with different fusion strategies to achieve two multimodality experiments: combine tongue image and chest CT, and combine tongue and chest X-rays. Fortunately, extensive repeated experimental results demonstrate the additionally using tongue images can improve the screening accuracy based on chest CT or X-rays. The results of the two multimodality experiments are reported as follows, respectively.

#### 4.3.1. The Fusion of Chest CT and Tongue Images

Table 4 reports the results on the screening of COVID-19-based single-modality CT data and the multimodality data (tongue image and chest CT).  Figure 8 shows the examples of incorrectly and correctly classified CT images. In summary, the multimodality model remarkably outperforms the single-modality model, which proves the feasibility of combining tongue images additionally. Specificity, for the chest CT classification task, we select out the modified AlexNet and ResNet50 to provide baselines. According to the results in Table 4, ResNet achieved a classification accuracy of 92.31%, and its sensitivity reached 92.34%. We also adopt different multimodality feature fusion strategies, including concatenation, add, and gated attention modules, to fuse tongue image features and CT features. As can be seen from Table 3, the multimodality classifier using the concatenation fusion strategy achieves the best classification results, and the accuracy of screening for COVID-19 reaches to 98.98%, which produces a significant improvement of 4.75% compared with the highest accuracy achieved by the single-modality model. At the same time, the classification accuracies of the other two fusion strategies significantly outperform the single-modality models.

When the tongue image is additionally used, the greatest change among the three evaluation metrics is specificity, but the accuracy and sensitivity also do change much. We analyzed that the sensitivity of COVID-19 to true negative categories increased when the tongue features were integrated into CT images, which helped reduce the additional examination to reduce the screening burden of suspected personnel and hospitals. From the perspective of three different fusion strategies, the concatenation strategy achieves the most considerable improvement. The reason is that tongue image and chest X-ray images belong to heterogeneous data. For heterogeneous data, the concatenation is the most suitable fusion strategy.

We dissect the strengths of the multimodality models.  Figure 9 presents the ROC curves of the screening of COVID-19 with and without using tongue images, which characterizes the robustness and stability of multimodality models. Specificity, compared to the single-modality CT-based model, the multimodality significantly increases the AUC value by 1.21%. The confidence level of the classifier has also been improved.  Figure 10 reports the confusion matrixes of four types of models. The improvement can also be clearly found. Combining tongue image and chest CT reduces two bad cases, which once verifies the importance of tongue images. Since CT images are the most widely-used radiological images in the current clinical screening of COVID-19, combining tongue images and chest CT can be widely promoted for achieving the accurate and large-scale screening of COVID-19 in clinical.

#### 4.3.2. The Fusion of Chest X-Rays and Tongue Images

Table 5 reports the results on the screening of COVID-19-based single-modality X-ray data and the multimodality data (tongue image and chest X-ray). We can see that the multimodality model also remarkably outperforms the single-modality model, which once demonstrates that using tongue images can improve the screening accuracy of COVID-19. This result verifies that tongue image can be used in clinical as a critical indicator for the screening of COVID-19. Specificity, in the single-modality results based on chest X-rays, AlexNet achieved the best results compared to ResNet50. Similarly, among different fusion strategies, the concatenation produces the best performance. The attention-gating fusion strategy performs similarly to concatenation, indicating that different fusion strategies have less impact on the multimodality screening of COVID-19. According to the ROC curves, as shown in Figure 4, and the confusion matrixes, as demonstrated in Figure 10, the single-modality models obtain pool performance compared to multimodality models. We also find that the classification probabilities of COVID-19 based on chest X-rays are improved after the tongue image feature is embedded. In clinical COVID-19 screening, due to chest X-rays' imaging characteristics, the application range of X-rays is not as extensive as CT. However, chest X-rays can reflect the lesion from the whole to a certain extent, and the operation is simple and easy to access in primary hospitals. Therefore, the fusion of chest X-rays and tongue images is an effective solution for screening COVID-19 in areas where medical conditions are scarce.

### 4.4. Analysis

#### 4.4.1. Noisy Robustness

While previous extensive results have verified the discriminative ability of tongue images on distinguishing COVID-19 and non-COVID-19, we provide a broader spectrum for more in-depth analysis by introducing noisy labels. Following the protocol in the pioneering work [45], we create corrupted counterparts on the above single-modality data of tongue images as follows. We make the label corruption to test the discriminative ability of tongue images under noisy environments. Label corruption uniformly changes the label of each image into another class with a probability of 10%.  Table 6 reports the screening results of COVID-19 based on noisy tongue images using several convolutional neural networks. We can see that the performance of the modified AlexNet does not decrease. The other deep neural networks have a small decrease in performance. These results demonstrate that the discriminative ability of tongue images has strong robustness and generalization. Therefore, tongue images can be used for the automated screening of COVID-19 in practice.

#### 4.4.2. *T*-test

We further perform statistical analysis to ensure that the experimental results have statistical significance. A paired *t*-test between the multimodality model (concatenation) and the single-modality model (AlexNet) based on chest x-rays is at a 5% significance level with a *P* value of 0.015. This analysis result clearly shows that the improvement from the multimodality model is noticeable. The *P* values between the multimodality model (concatenation) and the single-modality model (AlexNet) based on chest CT images are also at a 5% significance level, proving that tongue images can assist the automated screening of COVID-19. These analyses verify that our insight that introducing tongue images as a critical indicator for the clinical screening of COVID-19 is correct.

## 5. Conclusion

In this paper, we studied the widely concerning question: can tongue image assist the automated screening of COVID-19? Our answer is yes. To the best of our knowledge, this study is the first work to investigate the feasibility of tongue images on screening COVID-19, which is urgently demanding to stop the pandemic. Specificity, to verify the discriminative ability of tongue images, we designed several automated COVID-19 screening experiments based on tongue images. To confirm whether or not the tongue image can assist the COVID-19 screening based on radiographic images, we used three types of feature fusion strategies to construct multistream methods for the fusion of different features. Extensive experiments have verified the effectiveness of automated screening of COVID-19 based on tongue images, which is an underexplored but more realistic solution. In-depth analyses have revealed the effectiveness and potential of tongue image as a clinical tool to relieve radiologists from laborious workloads, contributing to the large-scale screening of COVID-19. Our studies provide a new perspective and a unique solution to the widespread automated detection of COVID-19. Our studies suggest that clinical experts should pay more attention to the comprehensive analysis of tongue images, especially Chinese medicine doctors. However, tongue screening also has some limitations. Tongue screening for COVID-19 is one-sided and nucleic acid monitoring has higher sensitivity and specificity. Tongue image is only a way to provide auxiliary diagnosis in a specific environment and cannot be used as a direct reference.

## Figures and Tables

**Figure 1:** Samples of different types of modalities: tongue image, chest CT, and chest X-rays.

**Figure 2:** The patient number of the training set, validation set, and test set for the three modalities, respectively.

**Figure 3:** The image number of the training set, validation set, and test set for the three modalities, respectively.

**Figure 4:** The distribution of severity degrees of the 17 COVID-19 cases in the test set. We can see that ordinary patients account for the majority.

**Figure 5:** Structure of dual-stream convolutional neural network with different fusion strategy.

**Figure 6:** Schematic of the attention gate (AG).

**Figure 7:** Confusion matrix of COVID-19 screening based on tongue images. We can see that both the classes of COVID-19 and non-COVID-19 have one bade cases.

**Figure 8:** Examples of incorrectly and correctly classified CT images. (a) represents incorrectly classified image. (b) represents correctly classified image.

**Figure 9:** ROC curves of CT and X-rays with and without using tongue image.

**Figure 10:** Confusion matrixes of CT-based and X-ray-based single-modality and multimodality classification.

**Table 1:** The comparison between related works of AI-based COVID-19 analysis.

Method	Type	Data	Task
[1]	Lesion patch	CT	COVID-19 screening
[2]	Lesion patch	CT	COVID-19 screening
[5]	Lesion patch	CT	COVID-19 screening
[6]	Lesion patch	CT	COVID-19 screening
[7]	2D slice	CT	COVID-19 screening
[8]	2D slice	CT	COVID-19 screening
[9]	2D slice	CT	COVID-19 screening
[4]	2D slice	X-ray	COVID-19 screening
[29]	Lesion patch	X-ray	COVID-19 screening
[31]	2D slice	X-ray	COVID-19 screening
[26]	3D scan	CT	Patient severity assessment
[27]	3D scan	CT	Infection area segmentation
[28]	3D scan	CT	Infection area segmentation

**Table 2:** The architecture of single-modality classifier.

Stages	Layer	Filter/stride/padding
Feature extraction	Con2d(3, 64) + ReLU	11 × 11/4/2
	MaxPool2d	3 × 3/2
	Con2d(64,128) + ReLU	5 × 5/1/2
	MaxPool2d	3 × 3/2
	Con2d(128,256) + ReLU	3 × 3/1/1
	Con2d(256,128) + ReLU	3 × 3/1/1

Propressive classifier	AdaptiveMaxPool2d (6,6)	
	FC(128 × 6 × 6,128) + ReLU	
	Dropout (*P* = 0.7)	
	FC(128,64) + ReLU	
	Classifier (64,2)	

**Table 3:** The screening results of COVID-19 based on tongue image using several convolutional neural networks.

Methods	ACC.	SEN.	SPEC.	MCC
AlexNet	0.9839	0.9897	0.9667	0.9911
Vgg16	0.9516	0.9688	0.9333	0.9732
GoogLeNet	0.9839	0.9897	0.9667	0.9911
DenseNet121	0.9678	0.9375	0.9333	0.9468
ResNet18	0.9677	0.9688	0.9667	0.9732
ResNet50	0.9839	0.9688	0.9667	0.9732

**Table 4:** Classification results in single-modality CT and multimodality data (tongue image and CT).

Modality	Classifier	ACC.	SEN.	SPEC.	MCC
Chest CT	AlexNet	0.9423	0.9091	0.8967	0.9232
	ResNet50	0.9231	0.9234	0.8667	0.9350

Multimodality	Concat	0.9898	0.9545	1.0	0.9611
	Add	0.9615	0.9545	0.9667	0.9212
	AG	0.9615	0.9545	0.9667	0.9212

**Table 5:** Classification results in single-modality X-rays and multimodality data (tongue image and X-rays).

Modality	Classifier	ACC.	SEN.	SPEC.	MCC.
Chest X-ray	AlexNet	0.9231	0.9545	0.9333	0.8832
	ResNet50	0.7692	0.8636	0.7000	0.8860

Multimodality	Concat	0.9808	0.9545	1.0	0.9611
	Add	0.9808	0.9545	0.9667	0.9212
	AG	0.9808	0.9545	1.0	0.9611

**Table 6:** The screening results of COVID-19 based on noisy tongue images using several convolutional neural networks.

Methods	ACC.	SEN.	SPEC.	MCC
Vgg16	0.871	0.781	0.9667	0.7361
GoogLeNet	0.9032	0.9688	0.8333	0.8142
DenseNet121	0.9355	0.9688	0.9	0.8720
ResNet18	0.9677	0.9375	1.0	0.9342
ResNet50	0.9514	0.9688	0.9333	0.9021
AlexNet	0.9839	0.9897	0.9667	0.9672

## Data Availability

The datasets generated for this study are available on request.
